This article has been retracted.

# A Comprehensive Nursing Model Combined with High-Quality Nursing Intervention for Antiviral Therapy in Patients with Chronic Hepatitis B

**DOI:** 10.1155/2022/6244637

**Published:** 2022-08-08

**Authors:** Wei Yang, Xiaofeng Tian, Jing Liang

**Affiliations:** ^1^Department of Hepatobiliary and Pancreatic Surgery, China-Japan Union Hospital, Jilin University, Changchun, Jilin, China; ^2^Department of Gastrointestinal and Colorectal Surgery, China-Japan Union Hospital of Jilin University, Changchun, Jilin, China

## Abstract

**Objective:**

To investigate the effect of comprehensive nursing combined with high-quality nursing intervention on the compliance, anxiety, and mental state of patients with chronic hepatitis B undergoing antiviral therapy.

**Methods:**

A total of 100 patients with chronic hepatitis B admitted to China-Japan Union Hospital from December 2017 to August 2020 were recruited and assigned to receive either routine nursing (control group, *n* = 50) or comprehensive nursing plus high-quality nursing (observation group, *n* = 50) via the random number table method. The outcome measures included compliance, psychological state, and treatment effects.

**Results:**

Before the nursing, there was no significant difference in the compliance scores between the two groups of patients (*P* > 0.05). After the nursing, the observation group had higher compliance scores than the control group (*P* < 0.001). Before the intervention, the two groups had similar Self-Rating Anxiety Scale (SAS) scores (*P* > 0.05). After the intervention, patients in the observation group showed lower SAS scores and a lower incidence of negative emotions as compared to the control group (*P* < 0.001). The observation group showed a better outcome in terms of quality of life, Medical Coping Modes Questionnaire (MCMQ) scores, and the General Self-Efficacy Scale (GSES) scores when compared to those of the control group (*P* < 0.001). A higher treatment effective rate was witnessed in the observation group in contrast to the control group (*P* < 0.001).

**Conclusion:**

The comprehensive nursing model combined with high-quality nursing intervention improves the psychological state and compliance of patients with chronic hepatitis B, with favorable treatment efficiency, which shows good potential for clinical promotion.

## 1. Introduction

Chronic hepatitis B (CHB) is a liver infectious disease caused by the hepatitis B virus (HBV) with high prevalence and contagiousness, long disease course, and frequent recurrence [1–3]. Long-term HBV infection is associated with liver cirrhosis and even hepatic cancer, posing potential health risks to patients [4]. Antiviral treatment of CHB provides long-term suppression of HBV and lowers the risk of complications with a promising therapeutic effect [5–7]. At present, the clinical antihepatitis B virus drugs include nucleoside analogues and interferons, of which nucleoside analogues are mostly adopted for long-term treatment, while interferons are used sparingly due to an inconvenient administration method (injection) and potential side effects. There are four antihepatitis B virus nucleoside analogues marketed for clinical use in China, namely lamivudine, telbivudine, entecavir, and adefovir, which are used to prevent or delay the adverse progression of chronic hepatitis B [8]. However, these drugs require long-term administration to consolidate the efficacy, and irregular use of the drugs is associated with drug resistance of the hepatitis B virus, resulting in complicated follow-up treatment. In addition, negative emotions during the long-term treatment may compromise the therapeutic effect [8–11]. To address such issues, effective nursing is recommended to enhance treatment compliance of patients and eliminate their negative emotions [12]. Comprehensive nursing refers to the systematization of nursing procedures and the coordination of nursing objectives, nurse responsibilities, evaluation, standardized nursing programs, health education, discharge management, and nursing quality control, while high-quality nursing highlights the rational arrangement of nursing staff and the efficiency of case handover to ensure the level and quality of nursing services. The combined application of the two nursing methods strengthens the overall nursing quality by incorporating the physiological, psychological, and social needs of patients into the objectives of nursing services [13–15]. The quality of life is an important prognostic indicator for CHB, and the combination of traditional Chinese medicine (TCM) with western medicine treatment can improve the antiviral efficacy and the quality of life of CHB patients.

Accordingly, this study investigated the effect of comprehensive nursing combined with high-quality nursing intervention on the compliance, anxiety, and psychology of patients with CHB to provide a new nursing direction for CHB patients. The report is as follows.

## 2. Materials and Methods

### 2.1. General Information

A total of 100 patients with chronic hepatitis B admitted to China-Japan Union Hospital from December 2017 to August 2020 were included.

#### 2.1.1. Inclusion Criteria

Patients who met the diagnostic criteria of chronic hepatitis B [16], without other serious organ diseases, with clear consciousness, normal hearing, no communication disorder, no limb movement disorder, without contraindications to nucleoside analogues, who received antiviral treatment for the first time, and who provided written informed consent were considered eligible.

#### 2.1.2. Exclusion Criteria

Patients with fatty liver, drug-induced liver injury, alcoholic liver injury, and other liver diseases, with hepatitis A, hepatitis C, hepatitis D, hepatitis E, AIDS, and other viruses, with hepatic and kidney dysfunctions, with allergies to drugs, infected with interferon, during pregnancy, and who have recently participated in or are currently participating in other clinical trials were excluded.

This study was approved by the Medical Ethics Committee of China-Japan Union Hospital, No.587 [11], and all subjects signed an informed consent form. According to the random number table method, they were divided into a control group and an observation group, with 50 cases in each group. Patients in the control group aged 24–70 years old, and those in the observation group aged 24–69 years old.

### 2.2. Research Methods

#### 2.2.1. Nursing Methods of the Control Group

Patients in the control group received routine care, which mainly includes routine monitoring of vital signs, monitoring of adverse reactions, medication compliance, and discharge instructions [10]. The patients' excreta were disinfected before disposal. Patients and their families were given health education about hepatitis B disease, antiviral treatment, transmission routes, and preventive measures to improve their awareness of the disease and treatment cooperation [11]. For example, chronic hepatitis B patients and other people's household items should be used separately, and the hepatitis B virus could be transmitted by breastfeeding. Dietary guidance was given as follows: patients were instructed to follow a high-protein, high-vitamin, low-fat diet, and were advised against stimulating, spicy, and cold foods, smoking, and alcohol [12]. Medication guidance was given as follows: patients were advised to follow the doctor's prescription strictly and should not change the type and dose of medication or suspend the treatment. The injection site was protected and the patients were reviewed regularly to prevent the development of drug resistance.

#### 2.2.2. Nursing Methods of the Observation Group

Patients in the observation group received comprehensive nursing combined with high-quality nursing. The specific measures are as follows:

1. Health education: (1) the patients were given CHB brochures and 30-minute lectures on CHB knowledge by professional doctors or nurses once a week to eliminate their negative emotions; (2) targeted one-to-one health knowledge lectures were given based on the patient's understanding to help them resolve issues about disease knowledge; (3) the health knowledge of CHB was also provided through education videos via the in-hospital multimedia equipment.
2. Medication nursing: (1) the patients received medication instructions, and changes in the dosage or the discontinuation of medication were prohibited; (2) before medication, the patients were instructed in terms of the objectives, methods, timing, dosage, precautions, contraindications, and possible adverse reactions of medication, and were informed of the importance of timely medication; (3) the clinical manifestations of the patients were closely monitored, and serious adverse reactions were reported to the doctor promptly for proper treatment.
3. Psychological nursing: (1) regular patient exchanges on CHB antiviral treatment were conducted; (2) the patients were provided with a clean and tidy ward environment; (3) the patients were encouraged to share their inner feelings with the nurses or their family members to obtain emotional support; (4) psychological counseling was also available for the patients to timely relieve their psychological burdens and negative emotions; (5) the nurses actively communicated with the patients to establish a good nurse-patient relationship; (6) cases with successful treatment were introduced to patients to eliminate their concerns.
4. Diet nursing: during hospitalization, the patients were given dietary guidance to ensure a clean, healthy, and nutritionally balanced diet, including light meals, food rich in dietary fiber, more fresh fruits and vegetables, low-cholesterol, low-fat, and low-salt food, no spicy food, no smoking, and no alcohol.
5. Exercise intervention: the patients were instructed to perform proper exercises, such as Tai Chi, yoga, slow walking, and other aerobic exercises
6. Prevention and nursing of complications: the patient's mental state and diet were closely monitored, and the changes in the patient's skin color, iris color, urine output, urine color, stool color, and stool shape were recorded in detail. Examinations of serum creatinine and CT were regularly carried out.
7. Discharge guidance: (1) on the day before discharge, the patients were given well-rounded explanations and instructions about medication, diet, and exercise after discharge, and were guided on effective self-nursing methods; (2) the patients were reminded of regular re-examination, including blood routine and CHB examination. TCM adjuvant therapy and Jianpi Huoxue decoction were also introduced to all patients. The ingredients include 30 g of Pseudostellariae Radix, 15 g of Atractylodis Macrocephalae Rhizoma, 15 g of Poria, 10 g of Sevenlobed Yam Rhizome, 30 g of fried Trionycis Carapax, 3 g of ground beetle, 18 g of Salviae Miltiorrhizae Radix et Rhizoma, 12 g of Broussonetiae Fructus, and 12 g of Semen Cuscutae. The abovementioned herbs were decocted in water for oral administration, one dose daily, with half a dose administered in the morning and half a dose in the evening. The duration of treatment was 48 weeks, with 24 weeks as one course of treatment.

### 2.3. Observation Indicators

#### 2.3.1. Treatment Compliance

During the follow-up, a compliance questionnaire for patients with CHB prepared by our hospital was used to evaluate the treatment compliance of patients. The evaluation domains included adequate medication dosage, timely medication, improved lifestyles, and regular postoperative re-examination.

1. Compliance Score: The options for adequate medication dosage and timely medication were set as no, occasionally, basically yes, and yes, with a score from 0 to 3 points. An improved lifestyle included 4 aspects before and after the nursing, namely, reasonable diet, regular daily schedule, proper exercise, and no smoking and alcohol, with a score from 0 to 3 points for each item and a total score from 0 to 12 points. Regular re-examination was set with 1 point for yes and 0 points for no.
2. Degree of Compliance: The total score for compliance was 0–16 points, with 0 points for poor compliance, 1–6 points for moderately poor compliance, 7–11 points for mediocre compliance, 12–15 points for good compliance, and 16 points for excellent compliance.
3. Compliance Improvement: Improved compliance indicated that the patient's total compliance score has improved by more than 50% compared to before the intervention. Moderate compliance indicated that the patient's total compliance score increased by 18%～49%. Low compliance indicated that the patient's total compliance score increased <18%.

#### 2.3.2. SAS Score before and after Intervention

The Anxiety Self-Rating Scale (SAS) was used to evaluate the anxiety state of the two groups of patients before and after the nursing intervention. Evaluation criteria were as follows: 50–59 points indicate mild anxiety; 60–69 points indicate moderate anxiety; 70 points and above indicate severe anxiety, with a full score of 100 points.

#### 2.3.3. Psychological Condition

The negative psychological conditions of the two groups of patients were recorded, including fear and anxiety due to illness, fear of infecting family members, fear of being alienated, fear of a poor prognosis, anxiety due to restricted mobility, and fear of disease recurrence.

#### 2.3.4. Quality of Life

The quality of life of the patients was evaluated according to the MOS 36-Item Short-Form Health Survey (SF-36), including physical functioning (PF), role physical (RP), bodily pain (BP), general health (GH), vitality (VT), social functioning (SF), role emotional (RE), and mental health (MH). The full score of each item is 100 points. The higher the score, the higher the quality of life.

#### 2.3.5. Comparison of Coping Mode and Self-Efficacy

The Medical Coping Modes Questionnaire (MCMQ) and the General Self-Efficacy Scale (GSES) were used to evaluate the quality of nursing in the two groups at admission and 4 weeks after nursing. MCMQ has a total of 20 questions covering three domains, namely, confrontation, avoidance, and yielding. The total score is 69 points. The higher the score, the greater the tendency in this aspect. GSES has 10 questions, and the patients are graded from 1 to 4 points corresponding to completely incorrect, somewhat correct, most correct, and completely correct, respectively. The higher the score, the higher the ability and self-confidence of patients to deal with the environment.

#### 2.3.6. Therapeutic Effect

The treatment effects include markedly effective, effective, and ineffective. Markedly effective: the HBV deoxyribonucleic acid (HBV-DNA) test showed a result within the normal range; effective: the HBV-DNA test showed a normal result with abnormal liver function indexes; ineffective: HBV-DNA and liver function indexes have not been improved. Treatment effective rate = (markedly effective + effective) number of cases/total number of cases × 100%.

### 2.4. Statistical Methods

SPSS22.0 statistical software was used to analyze and process the data in this study. The count data were expressed as *n* (%) and analyzed by the chi-square test; the measurement data were expressed as $\bar{x}$ ± *s*. Paired *t*-tests were used for intragroup comparisons and independent samples *t*-tests were used for intergroup comparisons. *P* < 0.05 indicates that the difference is statistically significant.

## 3. Results

### 3.1. Patient Characteristics

The baseline patient characteristics of the two groups were comparable (*P* > 0.05). (Table 1).

### 3.2. Comparison of Treatment Compliance

#### 3.2.1. Comparison of the Compliance Scores

Before the nursing intervention, there was no statistically significant difference in compliance scores between the two groups of patients (*P* > 0.05). After the nursing intervention, the observation group obtained higher scores of adequate medication dosage, timely medication, improved lifestyles, and regular postoperative re-examination than the control group (*P* < 0.001) (Table 2).

#### 3.2.2. Comparison of Compliance Degree

After the nursing intervention, the observation group had better compliance outcomes than the control group (*P* < 0.001), while the mediocre, moderately poor, and poor compliance rates, and the proportion of ineffective compliance were significantly lower than those of the control group (*P* < 0.001) (Table 3).

#### 3.2.3. Comparison of Compliance Changes

After the nursing intervention, in the observation group, there were 17 cases of improved compliance, 22 cases of moderate compliance, and 11 cases of ineffective compliance; in the control group, 8 cases of improved compliance, 10 cases of moderate compliance, and 32 cases of ineffective compliance. The observation group showed a higher proportion of improved and moderate compliance and a lower ineffective compliance rate than the control group (*χ*^2^ = 8.635, *P* < 0.05), as shown in Figure 1.

### 3.3. Comparison of Anxiety

Before the intervention, the two groups presented no significant disparity in SAS scores (*P* > 0.05). After the intervention, lower SAS scores were observed in the observation group, as compared to the control group (*P* < 0.001) (Table 4).

### 3.4. Comparison of the Psychological Conditions

The incidence of negative emotions including fear and anxiety due to illness, fear of infecting family members, fear of being alienated, fear of a poor prognosis, anxiety due to restricted mobility, and fear of disease recurrence in the observation group was significantly lower than those in the control group (*P* < 0.001) (Table 5).

### 3.5. Comparison of the Quality of Life

Before the intervention, the two groups showed no significant difference in the SF-36 scores (*P* > 0.05). After the intervention, the observation group had higher SF-36 scores when compared with those of the control group (*P* < 0.05), as shown in Table 6.

### 3.6. Comparison of Coping Mode and Self-Efficacy

In terms of the coping mode, the observation group yielded a significantly higher confrontation score, and lower scores of avoidance and yielding than the control group, indicating that patients in the observation group had better coping modes (*P* < 0.001 or 0.05). In addition, the GSES score of the observation group was significantly higher than that of the control group (*P* < 0.001). The results are shown in Table 7.

### 3.7. Comparison of Treatment Efficacy

There were 30 cases of markedly effective, 18 cases of effective, and 2 cases of ineffective in the observation group. There were 12 cases of markedly effective, 27 cases of effective, and 11 cases of ineffective in the control group. The overall treatment efficacy in the observation group (96.00%) was significantly higher than that of the control group (78.00%) (*χ*^2^ = 7.162, *P* < 0.05) (Figure 2).

## 4. Discussion

Patients with CHB are prone to negative emotions when undergoing antiviral therapy, and long-term negative psychological states may compromise the therapeutic effect [17]. Conventional nursing care is monotonous and inflexible and lacks relevance and humanistic care, resulting in frequent neglect of patients' psychological needs [18]. Therefore, a shift from purely therapeutic care to multifaceted care such as psychological, dietary, exercise, and health education is necessitated to enhance treatment compliance, reduce patients' negative emotions, and strengthen treatment efficacy [19]. Research has found that comprehensive care significantly improves the poor psychological status of elderly patients with perforated peptic ulcers [20], and high-quality care markedly improves treatment compliance and the condition of patients with chronic viral hepatitis with satisfactory results [21, 22]. Previous CHB treatment only emphasizes the efficacy and safety of drugs, but the growing demand of patients for high survival quality after CHB treatment has captured more clinical attention. It has been reported that TCM adjuvant therapy showed benefits in enhancing the survival quality of patients after CHB treatment, and the combination of Chinese and Western medicine may potentiate the clinical efficacy and improve the quality of life of patients [8]. The use of TCM prescriptions to strengthen the spleen and invigorate blood may strengthen the antiviral efficacy, but the specific mechanism requires further investigations. The results of this study showed significantly higher treatment compliance and treatment efficacy, and lower SAS scores and incidence of the negative psychological status of the patients in the observation group than in the control group after the nursing intervention, indicating that comprehensive nursing plus high-quality nursing contributes to enhancing the outcomes of CHB treatment from multiple facets, which may be attributed to the following reasons. The communications and interactions between patients during nursing helped patients maintain social relationships and share their feelings. The support from the family members and the nursing staff to the patients facilitated the establishment of a harmonious family relationship and patient-nurse relationship, thereby maintaining a positive and stable psychological status of the patients. Timely psychological counseling prevented the formation of severe mental issues in patients, and the introduction of cases with successful treatment outcomes enhanced their confidence against the disease. Disease-related health education corrected the patients' misunderstanding of CHB and enhanced patients' realization of the importance of active cooperation in treatment and self-care awareness, and the exercise and dietary instruction improved the patients' physical fitness and enhanced their immunity.

## 5. Conclusion

The comprehensive nursing model plus high-quality nursing intervention improves the psychological state and treatment compliance of patients with chronic hepatitis B, which shows great potential for clinical promotion.

## Figures and Tables

**Figure 1:** Comparison of compliance between two groups of patients. Note: after the nursing intervention, in the observation group, there were 17 cases of improved compliance, 22 cases of progressed compliance, and 11 cases of ineffective compliance; in the control group, 8 cases of improved compliance, 10 cases of progressed compliance, and 32 cases of ineffective compliance. The observation group was observed with a higher proportion of improved and progressed compliance and a lower ineffective compliance rate than the control group (*P* < 0.05).

**Figure 2:** Comparison of treatment effects between two groups of patients. Note: the results showed that in the observation group, 30 cases were markedly effective, 18 cases were effective, and 2 cases were ineffective; in the control group, 12 cases were markedly effective, 27 cases were effective, and 11 cases were ineffective. The overall effective rate of treatment in the observation group (96.00%) was significantly higher than that of the control group (78.00%) (*P* < 0.05).

**Table 1:** Comparison of general information between two groups of patients (*n* (%)).

Groups	Gender			Education level		
	Male	Female	Age (years)	Elementary school	Middle school or technical secondary school	Junior college and above
Control group (*n* = 50)	29 (58.00)	21 (42.00)	45.76 ± 8.49	9 (18.00)	27 (54.00)	14 (28.00)
Observation group (*n* = 50)	26 (52.00)	24 (48.00)	45.63 ± 8.42	8 (16.00)	25 (50.00)	17 (34.00)
*t*/*χ*^2^	0.364	0.077	0.426			
*P*	0.546	0.939	0.808			

**Table 2:** Comparison of compliance scores between two groups of patients ($\bar{x}$ ± *s*).

Timepoints	Groups	Adequate medication dosage	Timely medication	Improved lifestyles	Regular postoperative re-examination
Before intervention	Control group (*n* = 50)	1.66 ± 0.33	1.75 ± 0.39	5.97 ± 1.53	0.35 ± 0.13
	Observation group (*n* = 50)	1.64 ± 0.37	1.71 ± 0.42	6.02 ± 1.61	0.33 ± 0.10
*t*		0.285	0.494	0.159	0.862
*P*		0.776	0.623	0.874	0.391

After intervention	Control group (*n* = 50)	2.13 ± 0.31	2.04 ± 0.34	7.16 ± 1.83	0.49 ± 0.17
	Observation group (*n* = 50)	2.47 ± 0.35	2.58 ± 0.38	8.52 ± 2.19	0.67 ± 0.31
*t*		3.399	7.488	3.37	3.6
*P*		<0.001	<0.001	0.001	<0.001

**Table 3:** Comparison of compliance degree between two groups of patients after intervention (*n* (%)).

Groups	Excellent	Good	Mediocre	Moderately poor	Poor
Control group (*n* = 50)	7 (14.00)	13 (26.00)	11 (22.00)	9 (18.00)	10 (20.00)
Observation group (*n* = 50)	16 (32.00)	27 (54.00)	3 (6.00)	2 (4.00)	2 (4.00)
*χ* ^2^	4.574	8.167	5.316	5.005	6.061
*P*	0.032	0.004	0.021	0.025	0.014

**Table 4:** Comparison of SAS scores between two groups of patients ($\bar{x}$ ± *s*).

Groups	Before intervention	After intervention	*t*	*P*
Control group (*n* = 50)	57.04 ± 6.11	47.93 ± 5.74	7.684	<0.001
Observation group (*n* = 50)	57.81 ± 6.29	42.56 ± 5.18	13.230	<0.001
*t*	0.621	4.911		
*P*	0.536	<0.001		

**Table 5:** Comparison of psychological conditions between two groups of patients (*n* (%)).

Items	Control group (*n* = 50)	Observation group (*n* = 50)	*χ * ^2^	*P*
Fear and anxiety due to illness	23 (46.00)	13 (26.00)	4.340	0.037
Fear of infecting family members	43 (86.00)	18 (36.00)	26.272	<0.001
Fear of being alienated	36 (72.00)	12 (24.00)	23.077	<0.001
Fear of a poor prognosis	41 (82.00)	15 (30.00)	27.435	<0.001
Anxiety due to restricted mobility	40 (80.00)	14 (28.00)	27.214	<0.001
Fear of disease recurrence	38 (76.00)	11 (22.00)	29.172	<0.001

**Table 6:** Comparison of SF-36 scores between the two groups.

Groups	Before intervention	After intervention	*t*	*P*
Control group (*n* = 50)	52.39 ± 11.26	59.23 ± 11.25	3.309	0.003
Observation group (*n* = 50)	53.82 ± 9.26	66.26 ± 13.48	5.379	<0.001
*t*	0.694	2.831		
*P*	0.490	0.006		

**Table 7:** Comparison of coping mode and self-efficacy between the two groups of patients.

Groups	MCMQ			GSES
	Confrontation	Avoidance	Yielding	
Control group (*n* = 50)	28.29 ± 5.84	11.24 ± 3.14	6.12 ± 1.36	17.26 ± 3.73
Observation group (*n* = 50)	21.02 ± 6.48	13.18 ± 4.03	8.01 ± 2.36	24.28 ± 5.17
*t*	5.893	2.685	4.906	7.786
*P*	<0.001	0.009	<0.001	<0.001

## Data Availability

No data were used to support this study.
